The article "Expression of Matrix Metalloproteinase-9 in Gastric Cancer" was published in 2021. Journal: Cureus.

# Expression of Matrix Metalloproteinase-9 in Gastric Cancer

**DOI:** 10.7759/cureus.18195

**Published:** 2021-09-22

**Authors:** Prathipaa R, Priyathersini N, Thanka J

**Affiliations:** 1 Pathology, ACS Medical College and Hospital, Chennai, IND; 2 Pathology, Sri Ramachandra Institute of Higher Education and Research, Chennai, IND; 3 Pathology, Sree Balaji Medical College and Hospital, Chennai, IND

**Keywords:** collagenase, biomarker, matrix-metalloproteinase, mmp-9, gastric cancer

## Abstract

Background

Matrix-metalloproteinase-9 (MMP-9) is expressed by a wide range of cells and plays a significant role in the regulation of the tumor microenvironment of various cancers including gastric cancer. This study aims at the correlation of MMP-9 expression in gastric cancer with existing prognostic factors.

Methods

The MMP-9 expression in gastric cancer was identified by immunohistochemistry using a monoclonal antibody in paraffin-embedded sections, correlated with various clinicopathological parameters, and statistically analyzed.

Results

MMP-9 expression in gastric cancer was significantly correlated with the grade, depth of invasion, and TNM stage (p-value = 0.003, 0.019, and 0.025, respectively). A significant difference in expression between tumor tissue and adjacent gastric mucosa (p-value = 0.000) was also observed. 100% negative expression was found in well-differentiated tumors and early gastric carcinoma (T1).

Conclusion

The study results suggest that MMP-9 expression could be a potential biomarker of aggressive gastric cancer and candidates for the possible diagnostic and prognostic tool.

## Introduction

Gastric cancer is the malignant epithelial neoplasm that represents a biologically and genetically heterogeneous group of neoplasms with multifactorial etiologies. In the 1930s, gastric cancer was the leading cause of cancer-related death in the United States and Europe. Over the past 70 years, there is a dramatic decline in incidence and mortality in various parts of the world with the recent decline in non-cardia, intestinal type of adenocarcinomas, and a rising trend in proximal, diffuse-type adenocarcinomas in Western countries [1-3]. Currently, Gastric cancer ranks fifth most common cancer after lung, breast, colorectal, and prostate cancer worldwide. Gastric cancer is the third most common cause of cancer-related death worldwide in both sexes with 723,000 deaths annually. The highest estimated mortality rates are in Eastern Asia and the lowest in North America [4].

Matrix-metalloproteinases (MMPs) are a group of zinc-dependent enzymes present in the extracellular matrix of various tissues which plays a major role in the regulation of the tumor microenvironment. Among 23 human MMPs, MMP 2 and MMP-9 play a critical role in tumor invasion and angiogenesis because of their ability to degrade type IV collagen of basement membrane which forms the first barrier in the process of invasion, however, MMP-9 is 25 times more potent than MMP-2 [5]. MMP-9 is expressed by a wide range of cells including macrophages, neutrophils, and fibroblasts and its activity is regulated by cytokines, growth factors, and tissue inhibitors of matrix metalloproteinases (TIMP) [6]. MMP-9 also plays an important role in physiological conditions such as embryogenesis, tissue remodeling, and wound healing and pathological conditions such as inflammation, autoimmune diseases, and diabetes. It also plays an important role in immune cell function [7]. 

The article "Expression of Matrix Metalloproteinase-9 in Gastric Cancer" was published in 2021. Journal: Cureus.

Studies show increased expression of MMP-9 which is associated with invasion, metastasis, and poor prognosis in various cancers including cervical, colorectal, ovarian, and breast cancer [8-11]. In gastric carcinoma, overexpression of MMP-9 is correlated with increased metastatic potential, TNM staging, lymphatic invasion, depth of tumor invasion, and overall survival [12]. MMP-9 contributes to tumor metastasis via the sonic hedgehog signaling pathway in gastric cancer [13]. Its role in *Helicobacter pylori-*induced gastric inflammation, ulceration, and carcinogenesis were also observed [14]. The objective is to study the expression of MMP-9 (matrix metalloproteinase-9) in gastric cancer and to correlate it with the existing prognostic factors.

## Materials and methods

The study includes 100 gastric carcinoma cases of total and partial gastrectomy specimens from the Department of Pathology, in a Tertiary care center, collected during the time period between January 2015 and December 2019. The Institutional Ethical Committee in Sri Ramachandra Institute of Higher Education and Research approved the study (Ethics Committee Number: CSP-MED/15/JAN/21/01). The study parameters include age, sex, tumor size, site, differentiation status, lymphovascular invasion, depth of invasion (T), node (N) metastasis, distant metastasis (M), and TNM stage. The MMP-9 expression was studied and correlated with the study parameters.

The gastrectomy specimens were immediately fixed in 10% phosphate-buffered formalin for 24 to 48 hours. After gross examination, the representative bits from the tumor and adjacent normal tissue are submitted for processing using an automatic tissue processor. Paraffin sections of 5 µm thickness were made. Immunostaining of MMP-9 was done using 10 ml of ready to use IgG Rabbit Monoclonal (EP1255Y) Antibody to MMP-9 with 50 mg/ml of protein concentration. Section from bone marrow biopsy studied from 10 random individuals is used as positive control and cytoplasmic and nuclear staining of hematopoietic cells is regarded as positive for staining (Figure 1A). A negative control without the addition of a primary antibody is included in every batch of staining.

The article "Expression of Matrix Metalloproteinase-9 in Gastric Cancer" was published in 2021. Journal: Cureus.

**Figure 1:** Matrix metalloproteinase-9 expression in control, normal gastric mucosa, and gastric cancer (A) Control - bone marrow biopsy showing positive MMP-9 cytoplasmic and nuclear staining of hematopoietic cells, (B) normal gastric mucosa adjacent to tumor tissue show negative staining of MMP-9, (C) moderately differentiated gastric carcinoma with tumor cells showing positive MMP-9 cytoplasmic staining, (D) poorly differentiated gastric carcinoma with tumor cells showing positive MMP-9 cytoplasmic staining.

Assessment of MMP-9 expression in gastric carcinoma

At least 10 representative fields with maximum staining under high power magnification (400×) were chosen and 1000 cells were counted for each case. If the number of cells were less than 1000, then all the available cells were counted and results were expressed as a mean percentage. According to a study by Su-Zuan Chen et al. [15], cells exhibiting a brown-stained cytoplasm, at a higher intensity than the non-specific background staining were regarded as positively stained and tumors exhibiting positive staining in >10% of the total number of tumor cells were regarded as positive MMP-9 expression.

Statistical analysis

Statistical analysis was performed using Statistical Package for the Social Sciences (SPSS) software (IBM Corp., Armonk, NY). The Chi-square test was used for correlation between groups. Differences were assumed to be statistically significant if the p-value is <0.05.

## Results

Out of 100 cases of gastric carcinoma, 69% showed positive expression (Figure 1C-1D) and 31% showed negative expression. MMP-9 expression in tumor tissue (69%) was compared with adjacent gastric mucosa (15%) and a statistically significant difference was found (p-value=0.000; Figure 1B). The expression of MMP-9 was correlated with various clinicopathological parameters. MMP-9 expression increases with tumor differentiation. Out of 38 cases of poorly differentiated tumors 28 cases (73.7%) show positive MMP-9 expression (p-value = 0.003). MMP-9 expression increases with the depth of invasion (T), 18 out of 22 cases (81.8%) of T4 shows positive expression (p-value=0.019). MMP-9 expression shows a significant correlation with the TNM stage. Forty-nine cases are grouped in TNM stage III-IV, in which 39 cases (79.6%) show positive MMP-9 expression (p-value = 0.025). The mean age in our study is 58 years and the mean tumor size is 5 cm. Based on the mean age and tumor size, the cut-off value for the age and tumor size in our study is taken as 58 years and 5 cm, respectively. MMP-9 expression was observed more in age <58 years (35 out of 48 cases, 72.9%). The size of the tumor is ≥5 cm in 56 cases of which 73.2% show positive expression of MMP-9. The correlation of MMP-9 expression and clinicopathological parameters is summarized in Table 1.

The article "Expression of Matrix Metalloproteinase-9 in Gastric Cancer" was published in 2021. Journal: Cureus.

**Table 1:** Correlation of MMP-9 expression with clinicopathological parameters

Clinicopathological parameters	No of cases	MMP-9 + VE expression	P-value	Correlation
Age				
<58 years	48	35/48(72.9%)	0.416	Insignificant
≥58years	52	34/52(65.4%)		
Sex				
Male	68	48/68(70.6%)	0.617	Insignificant
Female	32	21/32(65.6%)		
Tumor size				
<5 cm	44	28/44(63.6%)	0.306	Insignificant
≥5 cm	56	41/56(73.2%)		
Tumor site				
Cardia	11	7/11(63.6%)	0.920	Insignificant
Body	20	14/20(70%)		
Antrum	69	48/69(69.6%)		
Histological types				
Intestinal	80	55/80(68.8%)	0.914	Insignificant
Diffuse	20	14/20(70%)		
Grade				
Well	5	0	0.003	Significant
Moderate	57	41/57(71.9%)		
Poor	38	28/38(73.7%)		
Lymphovascular invasion				
Present	52	36/52(69.2%)	0.959	Insignificant
Absent	48	33/48(68.7%)		
Primary tumor (T)				
T1	3	0	0.019	Significant
T2	47	16/47(59.3%)		
T3	48	35/48(72.9%)		
T4	22	18/22(81.8%)		
Lymph nodes (N)				
Positive	63	47/63(74.6%)	0.114	Insignificant
Negative	37	22/37(59.5%)		
Metastasis (M)				
M0	93	63/93(67.7%)	0.321	Insignificant
M1	7	6/7(85.7%)		
Stage				
Stage I-II	51	30/51(58.8%)	0.025	Significant
Stage III-IV	49	39/49(79.6%)		

## Discussion

MMP-9 is a zinc-dependent enzyme present in the extracellular milieu and involved in the regulation of the tumor microenvironment. The tumor-stromal crosstalk mediated by various cytokines and growth factors enhances the expression of MMP-9 which causes altered proteolysis. The key event is the degradation of the extracellular matrix - basement membrane of the epithelial cells which forms the first barrier in tumor invasion, cancer progression, and metastasis in gastric carcinoma making it more lethal and vulnerable. Our study shows 69% positive expression and 31% negative expression. MMP-9 expression is correlated with age, sex, tumor size, site, histological types, lymphovascular invasion, tumor differentiation, depth of invasion (T), lymph node (N) metastasis, distant metastasis, and TNM stage. A significant statistical correlation was seen with tumor differentiation, depth of invasion, and TNM stage (p-value =0.003, 0.019, and 0.025, respectively). In our study, increased MMP-9 expression was seen in cases with age <58 years (72.9%) and males (70.6%) which is in accordance with the study by Gao et al. in which 72.2% of cases with age <58 years and 76.2% of males show increased MMP-9 expression [16]. The average tumor size in our study is 5 cm and based on which tumor size is grouped into tumor size ≥5 cm (56 cases) and tumor size <5 cm (44 cases). The study observed increased expression in tumors ≥5 cm (41/56 cases, 73.2%). Body (14/20 cases, 70%) and antrum (48/69 cases, 69.6%) of the stomach show increased expression compared to the cardia. The study by Lee et al. found a significant correlation between Lauren histological types and MMP-9 expression with increased expression rate in intestinal-type [17]. However, our study shows increased expression in diffuse (14/20 cases, 70%) compared to intestinal (55/80 cases, 68.8%) type with no significant correlation. Our study shows increased expression in tumors with LV-invasion (69.2%). However, it is not statistically significant. In our study, we found increased expression in poorly differentiated tumors (28/38 cases, 73.7%) and 100% negative expression in well-differentiated tumors with statistically significant correlation (p-value=0.003). This shows that most of the poorly differentiated aggressive tumors show increased MMP-9 expression. The study by Zheng et al. shows significantly increased expression in advanced gastric carcinoma compared to early gastric carcinoma [18]. The study by Chu et al. [19] shows a significant correlation between depth of invasion and MMP-9 expression with increased expression rate in tumors with serosal invasion. Our study shows a statistically significant (p-value=0.019) increase in MMP-9 expression with a depth of invasion and maximum expression was seen in T4 (18/22 cases, 81.8%) and 100% negative expression in T1. This implies that most of the advanced gastric carcinoma and tumors with serosal invasion show increased MMP-9 expression. The study by Sun et al. shows a significant correlation between lymph node metastasis and MMP-9 expression and in our study lymph node-positive cases shows increased expression (47/63 cases, 74.6%) compared to lymph node-negative cases (22/37 cases, 59.5%). However, it was not statistically significant (p-value = 0.114) [20]. In our study, six out of seven cases with distant metastasis show MMP-9 expression (85.7%). The studies by Sun et al., Zheng et al., and Chu et al. show a statistically significant correlation between TNM stage and MMP-9 expression [18-20]. Our study also shows increased MMP-9 expression with TNM Stage III-IV (39/49 cases, 79.6%) compared to stage I-II (30/51 cases, 58.8%) tumors with statistically significant correlation (p-value = 0.025). This shows most of the tumors in the advanced TNM stage show increased MMP-9 expression. We also compared the expression of MMP-9 between tumor tissue and adjacent normal gastric mucosa in 100 cases. In our study, tumor tissue showed increased expression (69%) compared to adjacent gastric mucosa (15%) with a statistically significant correlation (p-value = 0.000).

The article "Expression of Matrix Metalloproteinase-9 in Gastric Cancer" was published in 2021. Journal: Cureus.

## Conclusions

MMP-9 present in the extracellular matrix plays a vital role in tumor invasion and progression of gastric cancer by acting as a key messenger between tumor cells, stromal cells, and cytokines which forms the tumor microenvironment. MMP-9 expression in gastric carcinoma is correlated with various histopathological parameters. MMP-9 expression is significantly increased in poorly differentiated gastric carcinomas, tumors with serosal perforation, and TNM stage III-IV tumors. These findings in our study suggest there is a significant role for MMP-9 expression in the depth of primary tumor invasion, grade, and TNM stage of gastric carcinoma.
